# Comparative proteomic analysis of membranous nephropathy biopsy tissues using quantitative proteomics

**DOI:** 10.3892/etm.2015.2197

**Published:** 2015-01-21

**Authors:** WEIGUO SUI, RUOHAN ZHANG, JIEJING CHEN, HUIYAN HE, ZHENZHEN CUI, MINGLIN OU, LI GUO, SHAN CONG, WEN XUE, YONG DAI

**Affiliations:** 1 Nephrology Department, Guilin 181^st^ Hospital, Guangxi Key Laboratory of Metabolic Disease Research, Guilin, Guangxi 541002, P.R. China; 2 College of Life Science, Guangxi Normal University, Guilin, Guangxi 541004, P.R. China; 3 Clinical Medical Research Center, The Second Clinical Medical College of Jinan University (Shenzhen People’s Hospital), Shenzhen, Guangdong 518020, P.R. China

**Keywords:** membranous nephropathy, proteome, isobaric tags for relative and absolute quantification, gene ontology analysis

## Abstract

Membranous nephropathy (MN) is a common cause of nephrotic syndrome in adults and the second leading cause of end-stage renal disease due to primary glomerulonephritis. The aim of the present study was to identify potential biomarkers of MN and further characterize these proteins by Gene Ontology (GO) analysis. Isobaric tags for relative and absolute quantification were used to compare the protein levels in tissues from MN patients and healthy individuals, and the combined samples were subsequently separated by specialized communications exchange. Mass spectrometry data acquisition was conducted using a 4800 Plus MALDI TOF/TOF tandem mass spectrometry device, and the results were subjected to statistical analysis. A total of 1,903 proteins were identified, with 423 proteins exhibiting a difference of >1.5-fold compared with the control group. Of these, 202 proteins were upregulated, while 221 proteins were downregulated. In conclusion, GO enrichment analysis revealed that the differentially expressed proteins were primarily mapped to the following GO terms: ‘Immune response’, ‘immune effector process’, ‘activation of immune response’ and ‘positive regulation of immune system process’. The affected proteins may be associated with the pathogenesis of MN; thus, may represent candidate MN biomarkers.

## Introduction

In adults, nephrotic syndrome is commonly caused by membranous nephropathy (MN), which is the second leading cause of end-stage renal disease (ESRD) due to primary glomerulonephritis (1). During the early stages of MN, IgG4 targets the M-type phospholipase A_2_ receptor. The IgG4 complex and/or other immune complexes are deposited on the subepithelial area of the basement membrane (2). A previous study estimated that one-third of MN patients develop ESRD or chronic renal failure and eventually require a renal transplantation (3). Although clinical manifestations, urinalysis, clinical chemistry tests and renal histopathology can be used to diagnose glomerular diseases, a renal biopsy provides a definitive diagnosis (4). Renal biopsy is an invasive procedure with the potential risk of serious complications, including hematoma, infection and arteriovenous fistula (5). Therefore, a safer and more effective diagnostic method is desirable. Biomarkers represent a potentially alternative method for diagnosis.

Proteomic technologies have enabled the identification of novel protein biomarkers (6,7). Technologies used for the discovery of protein biomarkers for glomerular diseases include two-dimensional (2D) gel electrophoresis, 2D differential in-gel electrophoresis, surface-enhanced laser desorption ionization time-of-flight (TOF) mass spectrometry (MS) and capillary electrophoresis-MS (4). Quantitative proteomic methods are used in the identification and quantification of proteins expressed at a genome-wide level or in a complex mixture (8). Isobaric tags for relative and absolute quantification (iTRAQ) is a technique developed by the Applied Biosystems Incorporation (8). Reagents used for iTRAQ consist of a peptide reactive group, a reporter group used in the analysis and a molecular mass balance group. iTRAQ is used to label samples with up to eight independent isobaric tags, which correspond to eight unique reporter ions (mass-to-charge ratio, 113–121). Therefore, quantitative information is obtained following integration of the peak areas for the eight different samples (8,9).

iTRAQ has been applied in the proteomic analysis of tissues from various diseases, including endometrial carcinoma (10), head and neck squamous cell carcinoma (11) and colorectal cancer (12). However, iTRAQ technology has been rarely used in the analysis of MN renal tissues. In the present study, iTRAQ was used to analyze the total protein content of renal tissues from patients with MN. The aim of the present study was to identify a safe, alternative, diagnostic method for MN, whilst improving the understanding of the mechanisms underlying the pathogenesis of MN.

## Subjects and methods

### MN and control groups

Renal tissue was collected from six MN patients between March and August 2011 at the Guilin 181^st^ Hospital (Guilin, China; Table I). The patients were diagnosed with MN through a biopsy, had a creatinine clearance level of ≥30 ml/min/1.73 m^2^ and suffered from persistent proteinuria of >5 g/24 h, although maximal tolerated angiotensin II was blockaded for at least four months (13). A renal biopsy was performed for all the patients with MN, and the results were examined by a certified pathologist in a blind analysis (the pathologist was unaware of the clinical and laboratory data). The control group consisted of only four individuals with normal kidney function and with no clinical evidence of MN, since normal renal tissue is difficult to collect and has a short storage life (Table I). Fig. 1 shows light photomicrographs (magnification, 200x) of the renal tissues from the MN patients, stained using hematoxylin-eosin and visualized under a microscopse (Nikon Coolscope II; Nikon Corporation, Tokyo, Japan). This study was performed according to the guidelines set forth by the Guilin 181^st^ Hospital and abides by the Declaration of Helsinki on ethical principles for medical research involving human subjects. Written informed consent was obtained from all the subjects or their guardians.

### Sample preparation

Biopsy samples were collected from the MN patients and control group. The samples were immediately washed with 0.9% RNase-free NaCl and briefly immersed in RNase inhibitor (Epicentre, Madison, WI, USA), according to the manufacturer’s instructions. The samples were stored at −80°C for subsequent analysis.

### Protein extraction and quantification

Renal tissue samples (250 mg) collected from the MN patients and control group were ground into a fine powder in liquid nitrogen, and supplemented with acetone. Subsequently, 10% trichloroacetic acid in acetone was added and the samples were incubated for 2 h at −20°C. Total protein was extracted using an extraction buffer, consisting of 8 M urea, 4% CHAPS, 40 mM Tris, 1 mM phenylmethylsulfonyl fluoride, 2 mM EDTA, 10 mM dithiothreitol and 0.5–2% isotonic glucose phosphate buffer (pH 8.5). Next, the samples were subjected to centrifugation at 40,000 × g for 1 h at 10°C. The protein concentration of the supernatant was determined using a bicinchoninic acid assay kit (Pierce Biotechnology, Inc., Rockford, IL, USA), according to the manufacturer’s instructions.

### iTRAQ reagent labeling, strong cation exchange (SCX) fractionation and tandem mass spectrometry (MS/MS)

Total protein in each group was pooled, blocked, digested and labeled according to the iTRAQ protocol (Applied Biosystems Life Technologies, Foster City, CA, USA). The iTRAQ tags were as follows: Healthy control, iTRAQ 113; MN, iTRAQ 119. The labeled digests were subsequently combined into one sample mixture.

Multidimensional liquid chromatography was performed to separate the tryptic peptides prior to MS. The combined samples were separated into ten SCX fractions using a 3.5-μm particle size column (35×0.3 mm, 300 Å; Zorbax Bio-SCX Series II; Agilent Technologies, Inc., Santa Clara, CA, USA) with a potassium formate gradient in 25% acetonitrile. The peptide fractions were further separated on a Tempo™ liquid chromatography nanoflow and matrix-assisted laser desorption/ionization (MALDI) spotting system (Applied Biosystems), equipped with a reversed-phase Magic C18Aq column (Applied Biosystems). Each chromatography run yielded ~380 MALDI spots on a stainless steel MALDI target plate (Applied Biosystems) (14).

A 4800 Plus MALDI TOF/TOF™ analyzer (Applied Biosystems Life Technologies) was used for MS data acquisition. Signal-to-noise ratios of ≥40 were required for MS/MS. Mass spectra from 500 laser shots were acquired for each spot. The MS/MS data from the ten SCX fractions were combined and analyzed using the Paragon Algorithm search engine and Human v3.62 (European Bioinformatics Institute, http://www.ebi.ac) (14).

### Statistical and Gene Ontology (GO) analyses

Proteins yielding tryptic peptides with average reporter ion ratios of ≥1.5 and ≤0.67 were classified as upregulated and downregulated, respectively. The GO database annotates selected proteins according to their molecular function (MF), cellular component (CC) and biological process (BP). To investigate the functions of the identified proteins, the online tool, Web Gene Ontology Annotation Plotting (http://wego.genomics.org.cn/), was used.

## Results

### Proteome of renal tissue

Using a peptide of >1 and a confidence interval of >95% (P<0.05) as the cutoff values for protein identification, a total of 1,903 proteins were identified and quantified from the collected renal tissues. Of the 423 proteins with >1.5-fold differences, 202 proteins were upregulated, while 221 proteins were downregulated. The beta-2-microglobulin level of MN was 1.56 times higher compared with the control group.

All the proteins were associated with the GO categories, MF, CC and BP. The most enriched MF terms included ‘protein binding’, ‘nucleotide binding’, ‘hydrolase activity’, ‘oxidoreductase activity’ and ‘nucleoside binding’ (Fig. 2). In addition, the most enriched CC terms included ‘intracellular’, ‘intracellular part’, ‘intracellular organelle’, ‘membrane-bounded organelle’ and ‘organelle part’ (Fig. 3). Finally, the most enriched BP terms included ‘cellular metabolic process’, ‘establishment of localization’, ‘transport’, ‘regulation of biological quality’ and ‘oxidation reduction’ (Fig. 4).

The upregulated and downregulated proteins belonging to the terms ‘immune response’, ‘immune effector process’, ‘activation of immune response’ and ‘positive regulation of immune system process’ are shown in Tables II and III.

## Discussion

The development of iTRAQ has enhanced the analysis of differential protein expression. Protein quantification using iTRAQ has been proposed as a suitable method for biomarker detection, since it permits parallel comparisons of protein abundance by measuring the peak intensities of reporter ions released from iTRAQ-tagged peptides. In the present study, iTRAQ technology and GO analysis were employed to perform quantitative proteomic analysis of plasma in MN tissue. A general proteome database was constructed for the renal tissue proteome, which has not been previously reported.

The use of GO proteomic analysis to investigate the observed changes was a necessary first step towards understanding the pathogenesis of MN. Differential proteins were assigned to the MF, CC and BP terms (Fig. 2–4), and GO enrichment analysis for the BP domain (Table III) revealed clusters of proteins for the following terms: ‘Immune response’, ‘immune effector process’, ‘activation of immune response’ and ‘positive regulation of immune system process’. Therefore, cellular and humoral immune mechanisms may play a major role in the pathogenesis of MN. By contrast, the subsequent progression to renal failure appears to be determined primarily by cell-mediated immunity. T-helper 2 (Th2) cells secrete a number of cytokines, including interleukin-4, -5, -10 and -13, which trigger B-cell activation and immunoglobulin synthesis. A previous study revealed that a predominance of Th2 cells may exist in MN patients, as shown by the presence of IgG, particularly IgG4 (15). This predominance complements deposits in the glomeruli and is a subclass of the type-2 immune response (15). B cell epitope spreading is a process whereby the primary immune response against the dominant initiating epitope further extends to other epitopes, either within the same molecule or among different molecules. This phenomenon may be relevant to the pathogenesis of membranous disease (16). Mesangial cells may contribute to the derangements occurring in MN, which have features of immune effector cells (17).

Beyond the observed upregulation or downregulation of protein expression, the proteins listed in Table II provide evidence that specific proteins in the kidney tissue may play an important role in MN. These results may facilitate the analysis of the role of these proteins in MN and support the proteomic study of the kidney tissue. A number of the identified proteins were mapped to the GO terms, ‘immune response’, ‘immune effector process’, ‘activation of immune response’ and ‘positive regulation of immune system process’. MN is considered to be an autoimmune disease, characterized by membrane-like thickening due to the accumulation of immune deposits on the outer glomerular basement membrane (16).

β_2_-microglobulin is a highly accurate and specific prognosis predictor; therefore, this parameter should be evaluated to avoid unnecessary immunosuppressive therapy (18). A previous retrospective study indicated that the urinary levels of β_2_-microglobulin and IgG are useful predictors of renal insufficiency in patients with MN (19). In the present study, β_2_-microglobulin was found to be highly expressed in the kidney tissues of MN patients (1.56 times higher compared with the control group), and was associated with the GO terms, ‘immune response’ and ‘positive regulation of immune system process’.

In conclusion, iTRAQ was used as a new strategy for proteomic analysis, and 1,903 proteins were found to be differentially expressed in the kidney tissues of MN patients when compared with the control group. GO enrichment analysis revealed that the differentially expressed proteins were primarily mapped to the GO terms, ‘immune response’, ‘immune effector process’, ‘activation of immune response’ and ‘positive regulation of immune system process’. The identified proteins may be associated with the pathogenesis of MN; thus, may be candidate biomarkers for the disease. However, these proteins require further verification.

## Figures and Tables

**Figure 1:** Images of renal tissue serial semi-thin sections from six patients with membranous nephropathy (hematoxylin-eosin; magnification, ×200).

**Figure 2:** Enriched Gene Ontology molecular function terms for membranous nephropathy tissue proteins.

**Figure 3:** Enriched Gene Ontology cellular component terms for membranous nephropathy tissue proteins.

**Figure 4:** Enriched Gene Ontology biological process terms for membranous nephropathy tissue proteins.

**Table I:** Main clinical and biochemical characteristics of patients with MN and the control group.

Characteristic	MN patients	Control group
Male/female, n	5/1	3/1
Age, years	47.17±12.17	39.52±17.23
Blood pressure, mmHg	143±26/75±12	122±12/73±11
Urinary protein excretion, g/24 h	6.7±3.45	-
Serum creatinine, mg/dl	1.21±0.52	-
Creatinine clearance, ml/min	73.54±29.75	-

MN, membranous nephropathy. −, within normal range (Urinary protein excretion, <0.15 g/24 h; serum creatinine, 0.15–1.2 mg/dl; creatinine clearance, 95–102±20 ml/min, where males had a value of 102±20 ml/min and females 95±20 ml/min).

**Table II:** Upregulated and downregulated proteins, belonging to the terms ‘immune response’, ‘immune effector process’, ‘activation of immune response’ and ‘positive regulation of immune system process’.

Uniprot accession no.	Protein name (Organism species = Homo sapiens)	Peptides (95% CI)	iTRAQ 119:113
Upregulated			
Q9NZP8	Complement C1r subcomponent-like protein (GN, C1RL; PE, 1; SV, 2)	1	2.3562
P07437	Tubulin β chain (GN, TUBB; PE, 1; SV, 2)	42	2.0528
P04233	HLA class II histocompatibility antigen γ chain (GN, CD74; PE, 1; SV, 3)	1	2.0146
P31146	Coronin-1A (GN, CORO1A; PE, 1; SV, 4)	5	1.5730
P61769	β_2_-microglobulin (GN, B2M; PE, 1; SV, 1)	4	1.5640
P04264	Keratin, type II cytoskeletal 1 (GN, KRT1; PE, 1; SV, 6)	46	1.5123
P52566	Rho GDP-dissociation inhibitor 2 (GN, ARHGDIB; PE, 1; SV, 3)	5	1.6968
P01911	HLA class II histocompatibility antigen, DRB1-15 β chain (GN, HLA-DRB1; PE, 1; SV, 2)	5	1.7591
P61769	β_2_-microglobulin (GN, B2M; PE, 1; SV, 1)	4	1.5640
P13746	HLA class I histocompatibility antigen, A-11 α chain (GN, HLA-A; PE, 1; SV, 1)	12	1.8167
Q9TQE0	HLA class II histocompatibility antigen, DRB1-9 β chain (GN, HLA-DRB1; PE, 2; SV, 1)	7	1.6628
P01857	Ig γ-1 chain C region (GN, IGHG1; PE, 1; SV, 1)	67	1.5854
P01594	Ig κ chain V-I region AU (GN, KV102; PE, 1; SV, 1)	4	1.6595
Q9NZ08	Endoplasmic reticulum aminopeptidase 1 (GN, ERAP1; PE, 1; SV, 3)	3	1.7790
Q96A32	Myosin regulatory light chain 2, skeletal muscle isoform (GN, MYLPF; PE, 2; SV, 1)	4	2.9194
P32455	Interferon-induced guanylate-binding protein 1 (GN, GBP1; PE, 1; SV, 1)	10	1.5951
P30481	HLA class I histocompatibility antigen, B-44 α chain (GN, HLA-B; PE, 1; SV, 1)	4	2.5680
P02794	Ferritin heavy chain (GN, FTH1; PE, 1; SV, 2)	6	2.0462
P19320-2	Isoform VCAM-6D of vascular cell adhesion protein 1 (GN, VCAM1)	3	1.6794
Downregulated			
P04003	C4b-binding protein α chain (GN, C4BPA; PE, 1; SV, 2)	1	0.5745
P10809	60 kDa heat shock protein, mitochondrial (GN, HSPD1; PE, 1; SV, 2)	47	0.5023
Q07021	Complement component 1 Q subcomponent-binding protein, mitochondrial (GN, C1QBP; PE, 1; SV, 1)	9	0.6528

GN, gene name; PE, protein existence; SV, sequence version; MN, membranous nephropathy; HLA, human leukocyte antigen; CI, confidence interval.

**Table III:** Proteins belonging to the specific biological process terms of the Gene Ontology enrichment analysis.

Term	Uniport accession no.
Immune response	P01031, P07437, P01876, P40306, P04003, Q9NZP8, P52566, Q07021, P30499, P01911, P61769, P01834, P13746, P28062, Q9TQE0, P01857, P04264, P63104, P31146, P01594, P02788, Q9Y3Z3, Q9NZ08, Q96A32, P04433, P01903, P04233, P10809, P05156, P32455, P30481, P13796, P02794
Immune effector process	P01903, P01031, P07437, P04233, P04003, P05156, P10809, Q9NZP8, Q9Y3Z3, P04264, P63104
Activation of immune response	P01031, P04003, P05156, P10809, Q9NZP8, P28482, P04264, P04216
Positive regulation of immune system process	P19320, P01031, P31146, P04003, Q9NZP8, P04216, P01903, P61769, P04233, P05156, P10809, P28482, P04264, Q08722
